# Three-Dimensional Ultrasound Images in the Assessment of Bladder Tumor Health Monitoring under Deep Learning Algorithms

This article has been retracted.

**DOI:** 10.1155/2022/9170274

**Published:** 2022-03-23

**Authors:** Changhua Shao, Aichun Sun, Hanwen Xue, Xianqiang Di

**Affiliations:** ^1^Department of Ultrasound, Tengzhou Central People's Hospital, No. 181 Xingtan Road, Tengzhou City 277599, Shandong Province, China; ^2^Department of Ultrasound, Zaozhuang Traditional Chinese Medicine Hospital, No. 2666 Taihang Mountain South Road, Xuecheng District, Zaozhuang City 277100 Shandong Province, China

## Abstract

This study was aimed at exploring the application value of three-dimensional (3D) ultrasound based on deep learning and continued nursing health monitoring (CNHM) mode in promoting the recovery of bladder cancer patients after surgery. 60 patients who underwent muscular noninvasive superficial bladder cancer and bladder perfusion treatment were selected as the research objects. The patients were randomly divided into two groups: an experimental group (30 cases) and a control group (30 cases). Patients in the experimental group adopted a CNHM model during the bladder perfusion treatment. The patients in control group adopted ordinary health monitoring mode. All patients underwent 3D ultrasound examination, and all images were processed using the convolutional neural network (CNN) algorithm. All patients were followed up regularly within 12 after the treatment. The imaging data, quality of life, satisfaction, and complications of the two groups of patients were compared in each time period. The ultrasound image processed by the CNN algorithm was clearer than that processed by the original method, showing higher image quality and more prominent lesion features. After 12 months of health monitoring intervention, the overall health status, scores of various functional areas, and score of functional subscales of the experimental group were greatly higher than those of the control group, and the differences were statistically significant (*P* < 0.05). The incidence of adverse reactions in the experimental group was much lower than that in the control group, and the difference was statistically obvious (*P* < 0.05). The comparison of the recurrence rate between the two groups of patients in each time period was statistically significant. The satisfaction score of the experimental group was much higher than the score of the control group, showing statistically significant difference (*P* < 0.05). CNN algorithm showed high application value in 3D ultrasound image processing, and the CNHM model was very beneficial to the postoperative recovery of bladder cancer patients.

## 1. Introduction

Bladder cancer is a malignant tumor with the highest incidence in the urinary system. In recent years, statistics from the World Health Organization show that the incidence of bladder cancer in developing countries has also shown an upward trend in the early years [1, 2]. Relevant research data show that the incidence of bladder cancer in China ranks 8th among malignant tumors and 1st among urinary system diseases [3]. Bladder cancer can generally be divided into two categories: nonmuscle invasive bladder cancer (NMIBC) and muscle invasive bladder cancer (MIBC). Among them, NMIBC is the most common, accounting for about 75%–85% of bladder cancer [4]. Regarding the treatment of bladder cancer, there are various treatment methods such as transurethral resection of bladder tumor (TUR-BT), transurethral laser surgery, and photodynamics [1]. At present, the most commonly used treatment method with better effect is transurethral resection of bladder tumor (TUR-BT). Although TUR-BT can completely remove the tumor, it has the problem of high recurrence rate [5]. Clinical studies have shown that the recurrence rate of bladder cancer after TUR-BT is as high as 50% within two years [6]. However, if you cooperate with bladder perfusion treatment after surgery, it can effectively reduce the recurrence rate of patients after surgery. At present, TUR-BT combined with postoperative bladder perfusion is the gold standard for the treatment of bladder cancer [7, 8].

Cystoscopy is the gold standard for the diagnosis and treatment of the bladder. However, as an invasive test, it often causes complications such as urethral injury and infection. In recent years, imaging technology has continued to develop. 3D ultrasound imaging technology can clearly show the details of bladder tumors. The detection rate of bladder cancer and the level of bladder cancer invading the bladder wall, namely T staging, have shown more and more advantages [9]. Ultrasound image reconstruction is a hot spot in the field of medical image processing in recent years. Among them, deep learning is an image processing algorithm that is widely used in the field of medical imaging [10]. Traditional learning algorithms have weaker feature expression ability due to the shallow training model, so their application in medical image feature extraction is limited. The depth learning algorithm is proposed under the background of advanced central processing unit, continuous improvement of machine algorithm, and massive medical images, which makes up for the shortcomings of traditional learning algorithms [1]. Research data shows that supervised deep learning algorithms have good effects and effects in the field of image analysis. In particular, the deep convolutional neural network (CNN) algorithm is currently the most valuable and potential method in the field of image processing and analysis [11].

In this work, bladder cancer patients were selected as the research objects, and the effects of continued nursing health monitoring (CNHM) mode on postoperative recovery were detected by ultrasound technology based on deep learning, aiming to provide reference and basis for clinical treatment and diagnosis of related diseases.

## 2. Research Materials and Methods

### 2.1. Research Objects

In this study, 60 patients who underwent muscular noninvasive superficial bladder cancer and bladder perfusion treatment in hospital from June 2019 to December 2020 were selected. The patients were randomly divided into two groups: experimental group (30 cases) and control group (30 cases). Among them, there were 33 male patients and 27 female patients. The average age of the patients was 64.3 ± 9.8 years old. This study had been approved by ethics committee of hospital and all subjects included in the study had signed the informed consent forms.

*Inclusion criteria*: patients who were diagnosed with muscular noninvasive bladder cancer according to the relevant diagnostic criteria of the *Guidelines for the Diagnosis and Treatment of Urological Diseases in China 2014*, with the surgical method of transurethral resection of bladder tumor (TUR- BT); patients in stable condition, with a clear mind and certain communication and understanding skills; and patients who can fill out the questionnaire smoothly.

*Exclusion criteria*: patients with complex bladder cancer or with complications of the kidney, brain, and heart; patients with serious infections that did not meet the indications for surgery; patients with cognitive impairment, poor communication skills, or mental disorders; and patients who were unwilling to participate in this study.

### 2.2. 3D Ultrasound Examination

The instruments included color Doppler ultrasound diagnostic apparatus, two-dimensional ultrasound imaging probe frequency, and 3D ultrasound imaging volume probe frequency of 5 ~ 7 MHz.

Before the examination, the patient was instructed to drink water. When the patient's urination was obvious and the bladder was full, it can perform routine ultrasound examination in the supine position to observe the tumor status. Then, it could use color Doppler ultrasound to observe the tumor blood flow signal distribution, use spectrum Doppler to measure hemodynamic parameters, and finally observe the level of tumor invasion of the bladder wall. During color Doppler ultrasound observation, it could start the 3D button on the basis of clearly displaying the two-dimensional ultrasound image, instruct the patient to hold their breath, and collect the image and store it. If it appeared, the image acquisition would be performed again. After the image acquisition is completed, the image is selected for 3D reconstruction (the reconstruction process is 3 ~ 5 s) and the reconstructed image of three axial planes (x, y, z) appears, then further adjustment was carried out, and the volume of the tumor was measured. The overall view of the tumor ultrasound image was selected for 3D reconstruction. It can start the slice key (3D tomographic imaging function) to perform 3D/CT, adjust the slice thickness and thickness interval of the slice as needed, and perform tomographic imaging of tumor lesions with a thickness of 1 mm on different axial planes.

### 2.3. Health Monitoring Methods

Patients in the control group underwent routine health monitoring. The first infusion time was 1 ~ 2 days before discharge. Health education was given for patients and their families before perfusion; the main content included disease-related knowledge, bladder perfusion knowledge, dietary knowledge, lifestyle knowledge, adverse reactions and prevention knowledge, psychological guidance, rehabilitation, and follow-up treatment guidance. At the same time, general patient information was collected. It should obtain the patient's phone number the day before discharge. The perfusion after discharge from the hospital was completed by the on-duty doctor, and relevant knowledge was propagated to the patient at the same time as the perfusion, and the next perfusion time was reserved at the same time. After 3 days of perfusion, the responsible nurse was responsible for telephone follow-up of the patient to collect information on complications, recurrence rate, quality of life, compliance, and adverse reactions. After 12 months of health monitoring, the satisfaction score would be performed.

Patients in the experimental group used the extended care model for health monitoring. The specific process was as follows: face-to-face on the first day after the surgery, the patient and his family members were taught about relevant knowledge, and general information about the patient was collected at the same time. Health education continued until the patient was discharged from the hospital to ensure that the patient understood and mastered the relevant knowledge of the disease and treatment. During this period, the patient was urged to act and develop good living habits. It can establish interactive platforms such as QQ, WeChat, and email before leaving the hospital. Within 12 months after the patient was discharged from the hospital, the patient was followed up by telephone within 3 days of the end of each chemotherapy treatment to assess the patient's psychological status, usual interactions, healthy behavior, living environment, and whether there were adverse reactions and corresponding measures. In addition, it can pass the latest health knowledge via phone, WeChat, QQ, email, etc., and give one-to-one health guidance and answers to questions for patients. The effect evaluation would be carried out after 12 months of health monitoring.

### 2.4. Image Processing Method

The deep CNN mainly includes four aspects: convolutional layer, pooling layer, fully connected layer, and Softmax classification layer. The calculation method of the convolution process was given as follows:

(1) $$\begin{array}{c} x_{j}^{l}=f\left(\underset{i\in M_{j}}{\sum }x_{j}^{l-1}•K_{ij}^{l}+{\text{b}}_{j}^{l}\right). \end{array}$$

In the above equation, *l* was the number of layers, *K* was the convolution kernel, *x*_*j*_^*l*−1^ referred to the feature map output by the previous layer, *K*_*ij*_^*l*^ represented the convolution kernel weight, *b* was the bias value, and *f*(•) was the activation function. The convolution operation contained three modes: Full convolution, Same convolution, and Valid convolution. The specific definitions were as follows:

The Full convolution was defined as below equation:

(2) $$\begin{array}{c} \left\{\begin{array}{c} y=conv\left(x,w,{}^{\prime }\text{ful}{\text{l}}^{\prime }\right)=\left(\text{y}\left(1\right),\cdots ,\text{y}\left(\text{t}\right),\cdots ,\text{y}\left(\text{n}+\text{m}-1\right)\right.\in \text{R}\\ y\left(\text{t}\right)=\overset{m}{\underset{i=1}{\sum }}x\left(\text{t}-\text{i}+1\right)•w\left(\text{i}\right)t=1,2,\cdots ,\text{n}+\text{m}-1 \end{array}\right.. \end{array}$$

The Same convolution was defined as equation (3):

(3) $$\begin{array}{c} \text{y}=\text{conv}\left(\text{x},\text{w},{}^{\prime }\text{sam}{\text{e}}^{\prime }\right)=\text{center}\left(\text{conv}\left(\text{x},\text{w},{}^{\prime }\text{ful}{\text{l}}^{\prime }\right),\text{n}\right)\in R. \end{array}$$

The Valid convolution was defined as equation (4):

(4) $$\begin{array}{c} \left\{\begin{array}{c} y=conv\left(\text{x},\text{w},{}^{\prime }\text{vali}{\text{d}}^{\prime }\right)=\left(\text{y}\left(\text{l}\right),\cdots ,\text{y}\left(\text{t}\right),\cdots ,\text{y}\left(\text{n}+\text{m}-1\right)\right)\in \text{R},\\ y\left(\text{t}\right)=\overset{m}{\underset{i=1}{\sum }}x\left(\text{t}+\text{i}-1\right)\text{w}\left(\text{i}\right)t=1,2\cdots ,\text{n}+\text{m}-1. \end{array}\right. \end{array}$$

The pooling layer can reduce the possibility of overfitting and improve the fault tolerance of the model. The expression equation of the pooling layer was as follows:

(5) $$\begin{array}{c} {\text{x}}_{j}^{l}=f\left(\beta_{j}^{l}\text{down}\left({\text{x}}_{j}^{l-1}\right)+b_{j}^{l}\right) \end{array}$$

In equation (5), down(•) was the down-sampling function and *β* and *b* were the multiplicative bias and the additive bias, respectively. There were two common pooling operations in convolutional neural networks: Mean pooling and Max pooling. Mean pooling was to output the mean value in the filter range as the pooling output. Maximum pooling was to use the maximum value in the filter range as a fully connected process of pooling output. In the convolutional neural network, the fully connected layer was a network node arranged linearly, and the output result of the previous layer was encoded into a one-dimensional vector. The fully connected layer was defined as follows:

(6) $$\begin{array}{c} {\text{x}}^{\text{l}}=f\left({\text{w}}^{\text{l}}{\text{x}}^{\text{l}-1}+{\text{b}}^{\text{l}}\right). \end{array}$$

In equation (6), w^l^ was the network weight coefficient, x^l−1^ referred to the output feature map of the upper layer, and b^l^ was the bias item of the fully connected layer.

Softmax classification layer was a multiclassifier connected to the fully connected layer. It can complete more than 2 types of classification tasks and convert multiple outputs into probability values in the (0,1) interval. In logistic regression, the training set was T = {(x^(1)^, y^(1)^), ⋯, (x^(m)^, y^(m)^)}, the input sample was x^i^ ∈ R^n^, and *y*^(i)^ referred to the sample label. If *y*^(i)^ ∈ {0, 1}, the hypothesis function could be defined by the following equation:

(7) $$\begin{array}{c} h_{\theta }\left(\text{x}\right)=\frac{1}{\left(1+{\text{e}}^{-\theta_{X}^{T}}\right)}. \end{array}$$

The cost function value J(*θ*) was minimized as the following:

(8) $$\begin{array}{c} \text{J}\left(\theta \right)=-\frac{1}{m}\left[\overset{m}{\underset{i=1}{\sum }}y^{\left(\text{i}\right)}\log{\text{h}}_{\theta }\left({\text{x}}^{\left(\text{i}\right)}\right)+\left(1-{\text{y}}^{\left(\text{i}\right)}\right)\log\left(1-{\text{h}}_{\theta }\left({\text{x}}^{\left(\text{i}\right)}\right)\right)\right]. \end{array}$$

The calculation equation of Softmax was shown as follows:

(9) $$\begin{array}{c} {\text{h}}_{\left(\theta \right)}\left({\text{x}}^{\left(\text{i}\right)}\right)=\left[\begin{array}{c} p\left(y^{\left(\text{i}\right)}=1\;|\;x^{\left(\text{i}\right)},\theta \right)\\ p\left({\text{y}}^{\left(\text{i}\right)}=2\;|\;{\text{x}}^{\left(\text{i}\right)},\theta \right)\\ \cdots \\ p\left({\text{y}}^{\left(\text{i}\right)}=\text{k}\;|\;{\text{x}}^{\left(\text{i}\right)},\theta \right) \end{array}\right]=\frac{1}{\sum_{j=1}^{k}e^{\theta_{j}^{T}x^{\left(\text{i}\right)}}}\left[\begin{array}{c} e^{\theta_{1}^{T}x^{\left(\text{i}\right)}}\\ e^{\theta_{2}^{T}X^{\left(\text{i}\right)}}\\ \cdots \\ e^{\theta_{K}^{T}x^{\left(\text{i}\right)}} \end{array}\right]. \end{array}$$

Learning on the training sample T minimized the damage function of Softmax. The expression of the minimum loss function was as follows:

(10) $$\begin{array}{c} \text{J}\left(\theta \right)=-\frac{1}{m}=\left[\overset{m}{\underset{i=1}{\sum }}\overset{k}{\underset{j=1}{\sum }}1\left\{y^{\left(\text{i}\right)}=\text{j}\right\}\log\frac{e^{\theta_{i}^{T}x^{\left(\text{i}\right)}}}{\sum_{i=1}^{k}e^{\theta_{i}^{T}x^{\left(\text{i}\right)}}}\right]. \end{array}$$

If 1{*y*^(i)^ = j} and *y* = *j*, the value was 1, or otherwise the value was 0. The smaller the loss function, the closer the month to the expected target.

### 2.5. Observation Indicators

The quality of life evaluation of patients mainly relied on the quality of life test scale for cancer patients (QLQ-C30) and the professional scale (QLQ-BLS24) for measuring the quality of life of patients with superficial noninvasive bladder cancer. The scale contained a total of 30 items, 15 fields, and 3 scales. The three scales included overall health status scale, function scale, and symptom scale. QLQ-BLS24 was a scale specifically for evaluating the quality of life of bladder cancer patients. The scale included 3 symptom subscales for bladder cancer patients, with a total of 24 items. The scale was scored using the Like4 score method: 1 point = no, 2 points = a little bit, 3 points = more, and 4 points = a lot.

The main items of the Doctor's Advice Behavior Evaluation Scale included 9 aspects: positive self-care attitude, uncomfortable symptoms and still perfusion, thinking that review and treatment were very important, regular review of treatment, abstinence from bad lifestyle habits, following doctor's advice and reasonable diet, regular review of cystoscopy, urine routine, regularly review liver and kidney function, pay attention to rest and sleep, and maintain emotional stability. The three-level scoring method was adopted: the possibility of accomplishing it was small, it was possible to do it, and it was completely accomplished, which were named as poor compliance with doctor's advice, good behavior with doctor's advice, and good behavior with doctor's advice. The corresponding score was 1 point ~3 points. The higher the score, the higher the patient's level of compliance behavior.

It should record the patient's bladder burning sensation, gastrointestinal reactions, urethral stricture, and urinary tract infection after each bladder perfusion.

The satisfaction evaluation scale was self-designed after consulting relevant experts. The satisfaction survey score was divided into 4 levels: very satisfied, satisfied, generally satisfied, and dissatisfied, which were counted as 3 points, 2 points, 1 point, and 0 points, respectively. The patient filled in the last perfusion to score the health monitoring service. The scale had been appraised by 3 nursing experts, and their recognition of the scale had reached 98%.

### 2.6. Statistical Methods

SPSS 22.0 statistical software was used for data analysis, and measurement data were expressed as mean ± standard deviation (x ± s). Comparison between groups was performed by t test, and comparison within groups was performed by analysis of variance. The count data was used by *χ*^2^ test and *P* < 0.05 meant the difference was statistically significant.

## 3. Results

### 3.1. General Data of Patients

The general information of the two groups of patients was shown in Table 1. Analysis of Table 1 shows that a total of 60 patients participated in this study, with 30 in the experimental group and 30 in the control group. There were 17 male patients and 13 female patients in the experimental group, with an average age of 64.8 ± 8.8 years old. There were 16 male patients and 14 female patients in the control group with an average age of 64.5 ± 8.1 years old. At the same time, two groups of patients had little difference in educational level, income, marital status, and other information. Therefore, the two groups of patients were comparable.

### 3.2. Comparison on Quality of Life Scores between the Two Groups of Patients Before and After Health Monitoring Intervention

The quality of life scores of the two groups of patients before and after the health monitoring intervention were shown in Figures 1 and 2, respectively. Analysis of Figure 1 shows that before the health monitoring intervention, the differences in overall health status, scores of various functional areas, and scores of functional subscales between the two groups of patients were not statistically significant (*P* > 0.05). After 12 months of health monitoring intervention, the overall health status, scores of functional areas, and score of functional subscales of the experimental group were significantly higher than those of the control group, and the differences were statistically significant (*P* < 0.05).

### 3.3. The Occurrence of Adverse Reactions in the Two Groups of Patients

After 12 months of intervention, the occurrence of adverse reactions of the two groups of patients was compared, as shown in Figure 3. In the experimental group, there were 1 case (3.3%), 2 cases (6.6%), 3 cases (10%), and 1 case (3.3%) with bladder irritation, urethral stricture, gastrointestinal reactions, and infections, respectively. In the control group, there were 3 cases (10%), 5 cases (16.6%), 6 cases (20%), and 5 cases (16.6%) with bladder irritation, urethral stricture, gastrointestinal reactions, and infections, respectively. The incidence of adverse reactions in the experimental group was much lower than that in the control group, and the difference was statistically significant (*P* < 0.05).

### 3.4. Comparison on the Number of Relapses After Bladder Perfusion Treatment between the Two Groups

During the treatment, the patients were followed up for a period of 12 months, and the postoperative recurrence of the two groups of patients was shown in Figure 4. The number of patients in the experimental group who relapsed after 3 months, 6 months, 9 months, and 12 months after surgery were 0, 1, 1, and 2, respectively, and those in the control group were 3 cases, 4 cases, 6 cases, and 5 cases, respectively. The difference in the recurrence rate between the two groups of patients in each time period was statistically significant.

### 3.5. Comparison of Compliance with Doctor's Orders between the Two Groups

Figure 5 shows the comparison of the two groups of patients' compliance with doctors after 12 months of health monitoring intervention. It illustrated hat the scores of the experimental group were significantly higher than those of the control group in the scores of compliance with the doctor's orders, and the difference was statistically significant (*P* < 0.05). This showed that the health monitoring method of the experimental group can significantly improve the patient's compliance behavior.

### 3.6. Comparison on Satisfaction Scores between the Two Groups of Patients After 12 Months of Intervention

The comparison of satisfaction scores between the two groups of patients after 12 months of intervention was shown in Figure 6. The satisfaction score of the experimental group was significantly higher than those of the control group, and the difference was statistically significant (*P* < 0.05). This suggested that the health monitoring method of the experimental group can significantly improve patient satisfaction.

### 3.7. Ultrasound Image of Typical Case

The ultrasound images of typical cases in the experimental group and the control group were shown in Figures 7 and 8, respectively. In the same time period, the 3D ultrasound showed that the patients in the experimental group recovered better than the control group. At the same time, comparison on the ultrasound images before and after revealed that the quality of the ultrasound images processed by the algorithm mentioned in this study was significantly improved, showing clearer images and more prominent lesion.

## 4. Discussion

Bladder cancer is the most common type of cancer in the urinary system. Its morbidity and mortality rank fourth among malignant tumors. Its incidence is relatively high in western developed countries, but its incidence in China has also been increasing in recent years. The ranking of malignant tumors in China has risen to the 8th place [12]. The disease can generally be divided into two categories: NMIBC and MIBC. Among them, NMIBC is the most common. Regarding the treatment of this disease, the most widely used clinically is TUR-BT. Although this method can completely remove the tumor, its recurrence rate is relatively high. Therefore, the clinical method of bladder perfusion is generally used to accompany the treatment. However, although bladder perfusion can significantly reduce the recurrence rate of bladder cancer, it has a longer treatment period and more complications. Therefore, it is difficult for most patients to persist, which affects the treatment effect and leads to bladder cancer recurrence. Therefore, it is very necessary to adopt certain health monitoring methods during treatment. At present, the commonly used clinical health monitoring methods for patients with malignant tumors are mostly technical and knowledge level and are often neglected for the mental health and guidance of patients [13]. It can be said that there are many shortcomings. In recent years, a CNHM model has gradually emerged in China and has been widely recognized. It has been widely used in the rehabilitation and health care of some chronic diseases, and has achieved good therapeutic effects. However, its application in the field of cancer health care is still less [14].

Regarding the diagnosis of bladder cancer, there are many diagnostic methods currently available. Cystoscopy, ultrasound, magnetic resonance imaging (MRI), CT and other techniques can all be used in the diagnosis of bladder cancer [15]. Although cystoscopy is the gold standard for diagnosis of bladder cancer, its use as an invasive test often causes various complications. CT examination may cover up the lesion due to insufficient bladder filling, and it also has the risk of exposing the patient to X-rays [16]. Although the accuracy of nuclear magnetic resonance is acceptable, the price is more expensive. With the continuous advancement of imaging technology, the accuracy of ultrasound diagnosis is further improved and its operation is simple and the price is relatively cheap. Therefore, it has been recognized by the majority of patients and doctors [17].

In recent years, computer and network technologies have continuously improved, and they have gradually penetrated into all aspects of people's lives. It has also been widely recognized and applied in the field of medical imaging [18, 19]. For example, the research and proposal of some computer-aided diagnosis systems and the application of computer technology in the segmentation of some tumor lesions [20]. One of the most concerned algorithms is the deep learning algorithm. It shows better performance in medical image processing, especially in image feature extraction. In recent years, deep learning algorithms have continued to advance and develop, and have been transformed and upgraded on the basis of the original algorithms. The CNN, a representative product of its development, has reportedly reduced the feature recognition error rate to 3.5%, and it can be said to be a very promising algorithm [21, 22].

In this study, a 3D ultrasound algorithm based on volume neural network was proposed and applied to the postoperative health monitoring effect of bladder cancer patients. It was found that the CNN had a better processing effect on ultrasound 3D images. The overall health status, scores of various functional areas, and score of functional subscales of the experimental group were greatly higher than those of the control group, and the differences were statistically significant (*P* < 0.05). The incidence of adverse reactions in the experimental group was much lower than that in the control group, and the difference was statistically obvious (*P* < 0.05). The comparison of the recurrence rate between the two groups of patients in each time period was statistically significant. The satisfaction score of the experimental group were much higher than the score of the control group, showing statistically significant difference (*P* < 0.05). Such results are consistent with previous studies.

## 5. Conclusion

In this study, a 3D ultrasound algorithm based on volume neural network was proposed and applied to the postoperative health monitoring effect of bladder cancer patients. It was found that the CNN had a better processing effect on ultrasound 3D images. Compared with the traditional health monitoring method, the CNHM mode was more conducive to the recovery of bladder cancer patients after surgery. The bladder cancer patients using CNHM were superior to ordinary health monitoring methods in terms of postoperative recovery, complications, and satisfaction. In this work, CNN algorithm and CNHM mode were introduced into the diagnosis and treatment of bladder cancer, providing a new idea and reference for the treatment and diagnosis of clinical related diseases. However, there were still some defects and deficiencies in this work. For example, it only analyzed the processing effect of one algorithm on 3D ultrasonic images and failed to introduce more new algorithms that attract more attention. In the future study and work, it will introduce more advanced algorithms to find the optimal image processing algorithm.

## Figures and Tables

**Figure 1:** The quality of life scores of the two groups of patients before the health monitoring intervention.

**Figure 2:** The quality of life scores of the two groups of patients after the health monitoring intervention. ∗Suggested that the difference was statistically obvious compared with the control group (*P* < 0.05).

**Figure 3:** Comparison on incidence of adverse reactions of patients. ∗Suggested that the difference was statistically obvious compared with the control group (*P* < 0.05).

**Figure 4:** Comparison on the recurrence rate of the two groups of patients during the postoperative period. ∗Suggested that the difference was statistically obvious compared with the control group (*P* < 0.05).

**Figure 5:** Comparison on compliance with doctor's orders between the two groups after 12 months of intervention. ∗Suggested that the difference was statistically obvious compared with the control group (*P* < 0.05).

**Figure 6:** Comparison on satisfaction scores between the two groups of patients after 12 months of intervention. ∗Suggested that the difference was statistically obvious compared with the control group (*P* < 0.05).

**Figure 7:** Ultrasound images before and after treatment in each time period of the experimental group.

**Figure 8:** Ultrasound images before and after treatment in each time period of the control group.

**Table 1:** Comparison on general data of patients.

Item		Experimental group (*n* = 30)	Control group (*n* = 30)
Age (years old)		64.8 ± 8.8	64.5 ± 8.1
Gender	Male	17	16
	Female	13	14
Education	Primary school	9	11
	Junior high school	8	10
	High school and above	13	9
Marital status	Unmarried, divorced or widowed	4	6
	Married	26	24
Occupation	On-the-job	7	10
	Retired	6	5
	Freelance	8	7
	Farming	9	8
Place of residence	Urban area	8	7
	Town	9	6
	Rural area	13	17
Medical payment method	New rural co-operative medical system	15	16
	Provincial and municipal employee medical insurance	13	11
	Own expense	2	3
Income	Below 1000 yuan	3	2
	1000–2000 yuan	11	12
	2000–3000 yuan	8	11
	3000 yuan and above	8	5

## Data Availability

The data used to support the findings of this study are available from the corresponding author upon request.
